# Optimization of Leach Protocol in Wireless Sensor Network Using Machine Learning

**DOI:** 10.1155/2022/5393251

**Published:** 2022-08-13

**Authors:** S. Ramesh, R. Rajalakshmi, Jaiprakash Narain Dwivedi, S. Selvakanmani, Bhaskar Pant, N. Bharath Kumar, Zelalem Fissiha Demssie

**Affiliations:** ^1^Department of Artificial Intelligence and Machine Learning, Saveetha School of Engineering, Saveetha Institute of Medical and Technical Sciences, Chennai, Tamil Nadu, India; ^2^Department of Computer Science and Engineering, Sathyabama Institute of Science and Technology, Chennai, Tamil Nadu, India; ^3^Department of Electronics & Communication Engineering, Engineering & Technology, Lingaya's Vidyapeeth, Faridabad, Haryana, India; ^4^Department of Information Technology, RMK Engineering College, RSM Nagar, Chennai 601204, India; ^5^Department of Computer Science and Engineering, Graphic Era Deemed to be University, Bell Road, Clement Town, Dehradun 248002, Uttarakhand, India; ^6^Department of Electrical and Electronics Engineering, Vignan's Foundation for Science Technology and Research, Guntur, India; ^7^Department of Computer Science, Ambo University, Ambo, Ethiopia

## Abstract

The Wireless Sensor Network is a network formed in areas human beings cannot access. The data need to be sensed by the sensor and transferred to the sink node. Many routing protocols are designed to route data from a single node to the sink node. One of the routing protocols is the hierarchical routing protocol, which passes on the sensed data hierarchically. The Low Energy Adaptive Clustering Hierarchy (LEACH) is one of the hierarchical methods in which communication happens in two steps: the setup phase and the steady-state phase. The efficiency of the LEACH has to be optimized to improve the network lifetime. Therefore, the *k*-means clustering algorithm, which comes under the unsupervised machine learning method, is incorporated with the LEACH algorithm and has shown better results. But the selection of cluster head needs to improvise because it will transfer the summed-up data to the sink node, so it is to be efficient enough. So, this paper proposes the modified *k*-means algorithm with LEACH protocol for optimizing the Wireless Sensor Network. In the modified *k*-means algorithm, the weight of the cluster head is tested and elected, and the clusters are formed using the Euclidean distance formula. The proposed work yields 48.85% efficiency compared to the existing protocol. It is also proven that the proposed work showed more successful data transfer to the sink node. The cluster head selection process elects the more efficient node as the head with less failure rate. The proposed work optimistically balanced the whole network in terms of energy and successful data transfer.

## 1. Introduction

The remotely controlled systems are greatly helping today's technology to grow. One such system is Wireless Sensor Network [1]. This network is formed by tiny sensors made to be in different positions in a scalable area. Those sensors are very tiny, battery-powered, and capable of gathering the information from their sensing area [2]. These nodes will communicate with each other through simple message exchanges. The sensors need to sense the information, transmit the gathered information, and request acknowledgement [3]. The data collected by nodes should be successfully transmitted to the central station for further processing [4]. This network's main usage is for forest, surveillance, aquaculture, mountain areas, etc. The transmission of information gathered and the usage of energy by the sensors are a very important parameter for increasing the lifetime of the Wireless Sensor Networks [5]. The resilience of the nodes or motes that have been used is an important criterion. The motes used may be movable or static. Many advancements are taking place in the hardware area of the sensor [6]. But proper protocols will help the sensors to transfer the data successfully and efficiently utilize energy for transferring and sensing the data. One such protocol is routing protocol, where the routing of information from one node to another and from nodes to central stations can take place following certain rules [7]. There are many routing protocols like data-centric routing protocol, hierarchical routing protocol, source-initiated routing protocol, destination-initiated routing protocol, location-based routing protocol, etc. [8]. Praveen Kumar et al. surveyed different machine learning methods used in the Wireless Sensor Networks for different purposes. Machine learning helps the sensor detect and send information according to the data sets already trained. So, machine learning schemes play a major role in Wireless Sensor Networks. All the routing protocols and many types of research were carried out in hierarchical protocols because it is a simple and economical way of processing the information [9].

Vishwakarma [10] discussed the principle of the LEACH algorithm which comes under the hierarchical routing protocol which has clusters formed in the scalable networks in which certain nodes will act as cluster heads, and other nodes will act as normal. The normal nodes collect information and transmit it to the cluster head. The cluster head will transmit the data gathered from all the nodes and send it to the central node [10]. Aziz and Arioua [11] used a hybrid *k*-means unsupervised algorithm in the clustered Wireless Sensor Network which trains the nodes with previous data collected and transmits the data from one cluster to another and so on [11]. The approach is for coordinating the movement of multiple sinks which are mobile through a central coordination point. To reduce the message overheads of storing the information of the prior sink movement path, they proposed another mechanism that proved to be energy efficient through simulations. The multiple MS path navigation algorithm for the multiple MS had maximum network coverage. The modified movement pattern was simulated and compared against existing protocols to prove the validity of the modified algorithm in terms of lifetime. A stable and energy-efficient data gathering approach uses mobile sinks for time-critical applications. According to the author, the speed at which the mobile sin moves is critical for data gathering for emergency applications. The modified protocol was validated by comparing it against competent protocols in the literature.

This research proposes the modified *k*-means unsupervised machine learning method in the LEACH routing protocol to enhance its life and optimize the network capacity.

## 2. Leach Routing Protocol

LEACH is the Low Energy Adaptive Clustering Hierarchical routing protocol. The main aim of this protocol is to keep the balanced weightage among all the nodes. It maintains the hierarchy by maintaining three members named sink, cluster head, and cluster nodes. The sink is the central station which receives the information from all the nodes and uses it for further processing [12]. The cluster head is the node randomly selected among the nodes with the criteria that it should not be selected more than once as a cluster head. This criterion is maintained to avoid the overloads for the same node once again. With its limited scalability, the cluster head selects the nodes within it. The cluster does this by sending the request messages to its nearby nodes. The nodes that send the acknowledgement back to the cluster head are added to its cluster. The cluster nodes play to sense the data from where it is deployed and transmit it to the cluster head, which goes to the sleep mode. The cluster head will wait for the information from all the nodes it added to its cluster network.

After receiving the information, the cluster head starts to aggregate the information and send the aggregated information to the sink node [13]. Few researchers conducted a detailed survey of the different mobility models in WSNs. The work proposed in this paper provided researchers with an insight into the available mobility models and their properties. According to the authors, each sink mobility model has its own properties. A categorization of the mobility models based on their general behaviour was also given in this paper. The basic categories mentioned are homogeneous mobility model and heterogeneous mobility model. Subcategories like controlled mobility, random mobility, totally and partially random mobility, predictable mobility, and geographic mobility were also mentioned.

Two phases occur in the LEACH protocol: the setup and steady-state phases. In the cluster head's setup phase, the cluster node's selection is made by the particular cluster head. In the steady-state phase, the transfer of information from the node to the cluster head and aggregated data from the cluster head to the sink node will occur [14]. The advantage of this LEACH protocol is a balanced workload among the nodes, fault tolerance, an easy and simple approach, an economical, easy manipulation process, etc. [15]. The main drawback of this approach is that the work in cluster head is overloaded because its capacity should be high enough to receive the data and send those data to the sink node; the cluster head will waste more energy if it is far away from the sink node; the cluster head is randomly selected which may not have enough energy to receive, aggregate, and transmit the data to the cluster head if the cluster head dies the information gathered by the nodes that are fully lost which leads to poor energy management; the overheated process will take place; the lifetime of the cluster head will reduce once it acts as the head; it may be exhausted fast, etc. [16]. Therefore, many advancements in the LEACH protocol were carried out differently. One of the best approaches is using machine learning algorithms in the LEACH protocol. Both supervised and unsupervised algorithms were used and studied. With the help of the data sets, the nodes are working smart and reducing the overhead.

## 3. Proposed LEACH Algorithm

This paper proposes a new method of using modified *k*-means machine learning with the LEACH routing protocol. The *k*-means algorithm is a grouping of elements based on the centroids calculated [17]. The centroids are calculated using Euclidean methods. The *k* number of the cluster is formed by categorizing the nearest value of the neighbours. At first, the points are selected randomly. Later using the iterative method, the centroids are found and the clusters are formed. It is quite simple to manipulate. In Wireless Sensor Network, *k*-means algorithms are used in the LEACH algorithm by forming clusters by choosing the cluster head with the help of centroids [18]. At first, the cluster head is chosen randomly by calculating the Euclidean distance and the cluster head is selected [19]. The selection of unsupervised learning is involved because the Wireless Sensor Network cannot be manipulated with the existing data set because the sensors are deployed only in the area where the human being is unaware.

In the proposed work, the cluster head is selected depending on the weightage assigned to the nodes. The weightage of the nodes is assigned according to the 'energy level of the particular sensor node. So the cluster head, along with the Euclidean distance, also has to satisfy the energy weightage. The cluster head is elected only if it is above the weightage parameter fixed. The main aim of fixing the weightage of the node is that it should be able to manage the work of the cluster head. The energy required to transmit the aggregated data needs to be calculated [20].

The energy required for the cluster head is

(1) $$\begin{array}{c} E_{\text{CH}}=n\left(k*\left(E_{\text{elec}}+E_{fs}\right.*d^{2}\right)\;\text{for }d<0,\\ E_{\text{CH}}=n\left(k*\left(E_{\text{elec}}+E_{\text{amp}}\right.*d^{4}\right)\;\text{for }d\geq 0. \end{array}$$

Here *E*_CH_ is the energy required by the cluster head*n* is the number of nodes assigned for the cluster, *k* is the number of message bits, *E*_elec_ is the energy required for sending and receiving the data bit, *£*_fs_ and *£*_amp_ are the parameter for calculating the *L*-bit message transmitting over free space multipath propagation, *d* is the transmitting distance towards the sink node.

The equation can represent the cluster head election using the *k*-means algorithm:

(2) $$\begin{array}{c} f=\sum_{c=1}^{m}\sum_{y\in g_{c}}{\left(y_{i}-h_{c}\right)}^{2}\;. \end{array}$$

*F* is the function of the *k*-means algorithm, *c* is the number of clusters, *y* is a mote of the cluster, and *h* is the head to be elected.

The Euclidean distance can be given by

(3) $$\begin{array}{c} d\left\{y_{i}\right),\left(\;h_{c}\right)={\left(y_{i}-h_{c}\right)}^{2}. \end{array}$$

*d* is the Euclidean distance of the nodes in the cluster.

In (2), the application of the *k*-means algorithm in the LEACH protocol is explained. Equation (3) tells the cluster formation using the Euclidean distance formula.

## 4. Results and Discussions

The proposed work is simulated using the parameters given in Table 1. The network area of 10000 m is taken where the 100 nodes were deployed. The initial node energy assigned to all the sensor nodes is considered 0.5 J. For the transmission and reception process, the sensor hardware needs 50 nJ energy [21]. The communication needs to be in free space or through multipath which is selected using the value *d*; accordingly, the value of *£*_fs_ or *£*_amp_ is selected. The energy consumed for the aggregation of data is taken as 5 nJ. With these parameters, the network is formed, and the connection between the nodes and the sink is established. Now, the LEACH algorithm is applied in the first round. From the second round, the cluster head was elected using the *k*-means algorithm, and weightage was calculated. Nearly 5000 rounds are simulated, and the nodes' energy is a routing protocol especially to reduce the energy consumption and balance the network energy. They used clustering and data filtering within the CHS. An application of the proposed protocol where the urban buses carry the mobile sinks was also explained [22]. This application was able to achieve maximum energy balance, connectivity, and throughput.

Figure 1 shows the simulation of the number of rounds versus the alive nodes. It is seen from the graph that simulation is taken for 5000 rounds for deployed 100 nodes. In the proposed work, after 950 rounds, the node energy is exhausted and dead. But in the existing protocol, the node death starts at 495 rounds itself [23]. The proposed work nodes are exhausted gradually compared to the existing algorithm. The presence of alive nodes is still 4555 rounds whereas for the existing algorithm, the system's total energy is exhausted at 2495 rounds itself. Figure 1 therefore proves that the proposed work enhanced the lifetime of the Wireless Sensor Network [24]. Therefore, the network's lifetime is increased by 45% compared to the existing algorithm. From Figure 1, it is seen that after 1000 rounds the alive nodes are decreasing but it is not the sudden fall as an existing method. In the proposed work due to the allowable loads given to the nodes, the work efficiency and the duration of life of every single node are increased. Therefore, the conclusion can be made that, due to iterations, training, and weightage factor, the energy of the whole network is optimally used. Therefore, the Wireless Sensor Network optimization is done through the proposed work. The cluster head selected based on its energy level helps all the nodes act as cluster head as well, and all nodes efficiently utilize its energy-packed up. It is seen that 48% of nodes were alive compared to the proposed work [25].

Figure 2 shows the simulation results of the number of rounds versus dead nodes for the proposed work. It is seen that it is the reverse calculation of Figure 1. The plot for this is to know the increase in the dead nodes during the number of nodes. From the analysis, it is seen that nearly 1 or none of the nodes were dead at many of the rounds. Approximately there is a depth of 5 to 6 nodes every 200 rounds after the death of the first node is calculated. Therefore, the node that acted as cluster head seems to be less dead. If the cluster head is not exhausted, the data collected from other nodes from the cluster are safely transmitted to the sink node [26]. Therefore, the energy weightage proposed helps the cluster save its energy for future use and prolong its lifetime in the network. The 100^th^ node death happened at 4555 rounds. Therefore, the whole network was actively working till 3000 rounds. After that, 25% of the nodes were dead, making the network efficiency a little less. Therefore, the proposed work optimized the whole network [27].

Figure 3 shows the simulation result of the number of rounds versus packets to the base station. Initially, 4000 bits were assigned for the node transmission. It is seen that nearly 310 kBps data were transmitted. Moreover, it is noticed that the data were successfully transmitted to the base station. Therefore, 77% of the data assigned to each sensor node were used and successfully transmitted to the sink node [28]. The cluster head selection with a good energy level plays a major role in successfully transmitting data packets. If the cluster head without sufficient energy was selected, it might not have the energy to aggregate and transmit data to the sink node. It leads to the loss of data and also the loss of the energy of the nodes present in that cluster [29]. Therefore, the proposed work optimally used all nodes and collected the sensed data efficiently [30]. The concept of BS mobility to extend the network lifetime provided theoretical results for the optimal movement of a BS where the transformation of the entire routing from the time domain to the space domain is given. An optimal period of the BS at specific points to increase the overall efficiency is found, and based on this, an approximation algorithm or routing was also developed [31].

The packets to BS are ten times the packets to the CH. This is because an average of 10 cluster heads will be elected in every round. Those ten cluster heads transfer data to the sink node. The problem related to the energy hole formation near the sinks was addressed by many researchers [32]. The energy holes near the sink partition the network and threaten the network's lifetime. The authors modified sink mobility to solve this problem [21]. They studied the network performance when the sink moves through predefined paths and stops at specific locations. This process achieved up to 4.86 times improvement in the network lifetime [33]. They also modified an algorithm wherein the sink can predict its next movement and presented simulation results to verify this approach [34].

Data delivery latency influenced the speed of the mobile sink. In a real-time scenario, mobile sink speed is restricted due to many factors. A solution for the same by choosing an optimal path as well as minimizing the energy consumption was proposed in this work. Theoretical analysis and simulation experiments were performed to validate the same in terms of energy consumption with existing algorithms [35].

Figure 4 shows the number of rounds versus the number of cluster heads elected. From the plot, it is seen that till the 1000 rounds, there were nearly 20 cluster heads elected for every round. After the 1000 rounds, the number of clusters elected is reduced and gradually decreases due to the reduction in energy level. It is also seen that the cluster head was present till 4500 rounds and after the cluster head selection is stopped. It shows that the nodes with proper weightage are only elected as cluster heads [36]. The nodes selected as cluster heads have sufficient energy to be elected, meaning nearly 10 nodes passed this threshold value in every round. Therefore, the node's energy was balanced, making it use its energy throughout the network lifetime [37].

Nearly ten nodes were elected as cluster heads in every round, which shows that all the nodes deployed in the network were given a role to act as cluster heads more than a time. A reliable and energy-efficient clustering algorithm was proposed by switching the roles of CHs, which focussed on predicting the CHs and controlling power levels. Balancing load among the sensors was also taken care of, leading to increased lifetime. They introduced a new formula for the probability of CH selection and the CH competition, which resulted in lifetime enhancement compared to LEACH. It gives an overview of the various energy-efficient clustering protocols. The authors highlighted the pros and cons of each protocol [35].

Figure 5 shows the number of packets to the cluster head versus several rounds. It shows the number of bits transmitted by the nodes to the cluster head for further transmission. It is seen that till 4000 rounds, 3.5 Mbps data packets were transmitted to all the nodes elected as cluster heads. Therefore, the cluster head efficiently used the *k*-means algorithm for forming the cluster and connecting the nodes to it. As the rounds increased, the data packets also increased gradually, showing the successful data transfer link between the cluster head and nodes. While using the proposed work, the cluster heads were effectively elected and the cluster head performed its role more efficiently. After aggregating and removing the same data obtained from the nodes, the cluster head transfers to the base station. If more cluster heads are elected, a greater number of clusters are formed, which leads to an overlap of information, and the energy of the nodes will get wasted. Therefore, the proposed work in every round approximately elects 10 cluster heads, forming nearly 10 clusters with nine nodes [38]. Therefore, it helps the cluster head efficiently form the network link and receive the data from the node in its Euclidean distance.

Figure 6 shows the plot of several nodes versus the energy consumption. It is known that 0.5 J energy is assumed for every node deployed. The above simulation is done for a single round. It is seen that nearly 10 microjoules of energy were spent by the whole every single round. Therefore, considering all the node's energy will be 50 J, only 10 microjoules of energy is spent in every round. Therefore, this is how the proposed work increased the network lifetime of the Wireless Sensor Network. Therefore, at 4000 rounds and total 50 joules of energy of all the nodes will be exhausted. It is seen that 10 microjoules of energy is used for a single round; therefore, for 4000 rounds, it will approximately come around 0.4 J of energy, equivalent to the energy of the nodes we assumed. Therefore, the proposed work optimistically manages the energy level of every node and enhances the lifetime of the Wireless Sensor Network. LEACH protocol for microsensor wireless networks provides ease of deployment, achieving maximum lifetime extension and latency and providing the application-specific quality. In LEACH, local computation is performed, reducing the overheads of data transmission, configuration, and operation of the network configuration. Experiment results showcased the high performance of LEACH in the constraints of the wireless environment.

Figure 7 shows the iterative result for the proposed work and the existing work. For 3 iterations, there were only 100 to 500 rounds of variation for the death of the first node. The iterative result therefore concluded that the proposed work obtained nearly 5% efficiency compared to the current work. The modified LEACH introduced an alternate CH replacement scheme and dual transmitting power levels. The performance of the modified MODLEACH was evaluated based on the parameters like throughput, formation of CHs and lifetime, and keeping hard and soft thresholds. The main aim of all the enhancements of the LEACH protocol is to increase energy efficiency.

## 5. Conclusion

The Wireless Sensor Network is optimized using LEACH protocol and a modified *k*-means algorithm. 48.85% efficiency has been obtained in terms of the lifetime of the network through the proposed work. The cluster head selection is also made in a balanced manner considering the nodes' energy. The packets to BS and packets to cluster head rate are increased using the proposed algorithm. The optimization between energy and the successful data transfer is very well maintained in this work. The overhead of the nodes is increased due to the addition of extra data regarding the energy of the nodes. It has increased the data bits usage. The sink node work also increased during the election of the cluster head. The cluster head was elected till the end of the lifetime of the whole network, which shows that the overall energy consumption is well maintained. Nearly 77% of the data sensed were transmitted to the sink node. The processing time of the *k*-means algorithm is increased due to the extra addition of the threshold value of the energy. It needs to be optimized in further work. The node's overhead increases due to the extra addition of energy status and the request message. The *k*-means algorithm increases the processing time for completion of the election of cluster head.

## Figures and Tables

**Figure 1:** Number of rounds versus alive nodes.

**Figure 2:** Number of rounds versus dead nodes.

**Figure 3:** Rounds versus packets to BS.

**Figure 4:** Rounds versus number of cluster heads elected.

**Figure 5:** Rounds versus packets to CH.

**Figure 6:** Number of nodes versus energy consumption.

**Figure 7:** Iterative results for the proposed work.

**Algorithm 1:** LEACH protocol Algorithm.

**Table 1:** Simulation parameters.

Simulation values	Values
Network area	100*∗*100 m
Position of the BS	(50, 50)
Number of nodes deployed	100
Initial node energy	0.5 J
Message size	4000 bits
Number of rounds	5000
Transmission amplifier free space, *£*_fs_	10 pJ/bit/m^2^
Transmission amplifier multipath, *£*amp	0.0013 pJ/bit/m^4^
Transmitting energy	50 nJ
Receiving energy	50 nJ
Aggregated data energy	5 nJ/bit/msg

## Data Availability

The data used to support the findings of this study are included within the article. Should further data or information be required, they are available from the corresponding author upon request.
